The article "Accounting Earnings and Economic Growth, Trends, and Challenges: A Bibliometric Approach" was published in 2022. Journal: Comput Intell Neurosci.

# Accounting Earnings and Economic Growth, Trends, and Challenges: A Bibliometric Approach

**DOI:** 10.1155/2022/7352160

**Published:** 2022-08-10

**Authors:** Mu Sun, Elena Urquía-Grande, Julián Chamizo-González, Cristina del Campo

**Affiliations:** ^1^Faculty of Economics & Business, Department of Financial Administration and Accounting, Complutense University of Madrid, Madrid 28223, Spain; ^2^Faculty of Economics & Business, Department of Accounting, Autonomous University of Madrid, Madrid 28049, Spain; ^3^Faculty of Economics & Business, Department of Financial and Actuarial Economics and Statistics, Complutense University of Madrid, Madrid 28223, Spain

## Abstract

In recent years, studies have been conducted to quantify the relationship between microeconomic and macroeconomic development. Macroeconomics is the orientation of microeconomic development. Existing research hopes to quantify the relationship between macroeconomics and micro-firms, rather than just focusing on economic indicators. And some empirical studies try to use the relationship between them to discuss its usefulness for micro-firm decision-making. This article focuses on applying and developing aggregate earnings in connecting microenterprise earnings and macroeconomic development. To achieve this goal, this research did a comprehensive bibliometric analysis on macro-accounting on the two most influential databases, namely, Web of Science and Scopus. It used the information visualization software VOSviewer to draw knowledge maps to sort research lines. We also analyzed the research hotspots of macro-accounting in recent years according to the year scale and combined it with the neural network PSO-LSTM model to predict their future development. It turns out that the research on aggregate earnings related to economic growth has become a research hotspot in recent years. Scopus research and development potential is better than Web of Science in this field.

## 1. Introduction

Since the 2008 global financial crisis, economies worldwide have experienced tremendous turbulences. When the world economy had not yet emerged from the shadow of the economic crisis, a new crisis had already arrived. The global pandemic of COVID-19 has worsened the already fragile global economic situation. The International Monetary Fund (IMF) report noted that the pandemic outbreak had affected global supply chains, exacerbating inflation in many countries [1].

Researchers have long valued the usefulness of accounting information in microeconomics. The theories of the usefulness of accounting for decision-making are critical. They do constitute the theoretical basis of the conceptual framework not only of the International Financial Reporting Standards (IFRS) in Europe but also of the Financial Accounting Standards Board (FASB) in the United States, applied all over the world [2].

The article "Accounting Earnings and Economic Growth, Trends, and Challenges: A Bibliometric Approach" was published in 2022. Journal: Comput Intell Neurosci.

In September 2010, the FASB and the IASB jointly issued Concept Statement No. 8 [3], replacing the original concept statement of Corporate Financial. This new statement determines that the financial reporting objective provides valuable financial information about the reporting entity. In IAS 1 latest revision [3], it was also noted that the purpose of financial reporting is to provide investors with more helpful information. In today's complex and changeable economic background, the study of accounting information is more practical. Existing related research mainly focuses on the research of accounting information for investors, creditors, and individuals [4–8]. However, at the macrolevel of the economy, there is a lack of research from an accounting perspective [9, 10].

This article aims at using mathematical and statistical methods to quantitatively analyze all knowledge carriers, that is, the bibliometric analysis method, to explore the relationship between microenterprise financial information and macroeconomy. Hence, this research aims at realizing a bibliometric analysis of the existing literature on accounting earnings that affect economic growth to find out the internal relationship between them. Moreover, this research hopes to predict the future development trend of this topic through the neural network model.

We also evaluate this research topic status in the scientific community in this emerging research direction. Therefore, the present research aims to provide a reference for research on the relationship between accounting information and macroeconomics and provide essential data for advancing future research in this field. The organization of this article is as follows. First, we outline the sources of research data and research methods. Secondly, we conduct a bibliometric analysis of the obtained literature data and discuss the results. Finally, main conclusions, limitations, and further research opportunities are defined.

According to the research objective of this article, the research question is defined as follows:

(RQ1) What is the development status of the existing research on accounting earnings and economic development?
(RQ2) What research trends will the research on accounting earnings and economic development have in the future?

## 2. Methodology

### 2.1. Research Field and Databases

This article explores the current research status of microenterprise financial information and economic development trends. Fortunately, we found that this topic is one of the research lines of “usefulness of earnings” and the used indicator is usually the “aggregate earnings” of microenterprises. Therefore, we started by studying the usefulness of earnings and systematically exploring the development of this topic.

The article "Accounting Earnings and Economic Growth, Trends, and Challenges: A Bibliometric Approach" was published in 2022. Journal: Comput Intell Neurosci.

We use Scopus and Web of Science (WoS), as they are the primary sources for indexing scientific papers and collecting data from many articles. Both databases can provide reliable and high-quality literature search results [11]. We hope to compare and analyze the results of the two databases in this study. Integrating multiple databases to analyze scientific data can provide more reliable bibliometric analysis results [12].

Also, this article considers Price's law to explain the current research status better. Price [13] noticed in his research that there are always a few people who dominate publications within a topic. From this, he developed Price's law. According to Price's law, the four scientific research stages are the precursor stage, the exponential growth stage, the consolidation of the body knowledge stage, and the decrease in the production stage.

Accounting information is closely related to economic development, because accounting is one of the important tools for cost-effective economic development. Therefore, this article aims at investigating the research field of accounting information and macroeconomics. As pointed out above, the indicator “aggregate earnings” best represents this topic. However, due to the scarcity of existing literature, we started investigating from this topic's previous dimension—the research on the usefulness of earnings, using the keywords “usefulness” and “earnings” to search for keywords, abstracts, and topics. As for the “aggregate earnings” research line, although the literature is scarce, we have conducted an independent investigation.

### 2.2. Bibliometric Analysis

After completing the above preparations, this article will use the collected data for bibliometric analysis. Bibliometric analysis results can help us understand the research ability and the academic community's different research directions on this topic.

In this section, based on our findings on this topic, we will analyze the research lines' details of the usefulness of earnings in this section according to what we have discovered about this topic. We will also use the information visualization software VOSviewer (Vision 1.6.7 for Microsoft Windows 11) to draw the corresponding knowledge maps based on the two databases' output (Scopus and WoS). It concentrates in a few lines the description of the expected results after using the software. The term co-occurrence map drawn by it can display the research trend changes on the time axis to understand the past and the latest research hot areas, and it can clearly show the existing research lines. Then, we will analyze the two databases' outputs and compare the similarities and differences to analyze the research status. Finally, the neural network model will predict future research hotspots of aggregate earnings topic in the two databases.

The article "Accounting Earnings and Economic Growth, Trends, and Challenges: A Bibliometric Approach" was published in 2022. Journal: Comput Intell Neurosci.

### 2.3. The Launch of the Deep Neural Network Model

The present research also wants to compare the predictive ability of traditional time series modeling ARIMA and neural network BP model and optimized PSO-LSTM model on this topic. For the ARIMA model, the differential moving average autoregressive model is referred to as the ARIMA model for short. It is mainly used to fit time series with stationary attributes or converted into a time series with stationary attributes. Box et al. [14] proposed the complete process of constructing an ARIMA model. The central idea is to make the unsteady original sequence stable through the difference operation method, where d is the total number of different operations; that is, by comparing the size of two fractions, it is difficult to solve by other quick methods such as “direct division” or “sameness.” The basic principle is as follows:

(1) $$\begin{array}{c} \varphi \left(A\right)\nabla^{d}x_{t}=\theta \left(A\right)\varepsilon_{t},\\ Q\left(\varepsilon_{t}\right)=0,\text{var}\left(\varepsilon_{t}\right)=\sigma_{\varepsilon }^{2},Q\left(\varepsilon_{t},\varepsilon_{s}\right)=0,\;s\neq t,\\ Q\left(\varepsilon_{t},\varepsilon_{s}\right)=0,\;\forall s<t. \end{array}$$

In the formula, ∇^*d*^=(1 − *A*)^*d*^, *φ*(*A*)=1 − *φ*_1_*B* − ⋯−*φ*_*p*_*B*^*p*^, *θ*(*A*)=1 − 1 − *θ*_1_*B* − ⋯−*θ*_*p*_*B*^*p*^ are the autoregressive polynomial coefficient and the moving smoothing polynomial coefficient of the stationary reversible ARIMA model, respectively. After unfolding the recurrent neural network, it can display the specific structure of the recurrent neural network. The forward propagation derivation formula is

(2) $$\begin{array}{c} a_{k}^{t}=\sum_{h=1}^{H}w_{hk}b_{h}^{t}, \end{array}$$

(3) $$\begin{array}{c} a_{k}^{t}=\sum_{i=1}^{I}w_{ih}x_{i}^{t}+\sum_{h^{\prime }=1}^{H}w_{h^{\prime }h}b_{h^{\prime }}^{t-1}, \end{array}$$

(4) $$\begin{array}{c} b_{h}^{t}=\theta_{h}a_{h}^{t}. \end{array}$$

In formulas (2)–(4), *b* represents the value calculated by the activation function, *a* represents the value calculated by the collection, and *w* is the parameter connected between different nodes. The output layer is subscripted *k*, the hidden layer is subscripted *h*, and all functions with parentheses. Both are activation functions. *ϵ* and *δ* are defined in the formula, and *L* is the final loss function. The specific calculation method is not written here because it is the same as the traditional BP neural network:

(5) $$\begin{array}{c} \delta_{h}^{t}=\theta^{\prime }\left(a_{h}^{t}\right)\left(\overset{K}{\underset{k=1}{\sum }}\delta_{k}^{t}w_{hk}+\overset{H}{\underset{h=1}{\sum }}\delta_{h^{\prime }}^{t+1}w_{h^{\prime }h}\right), \end{array}$$

(6) $$\begin{array}{c} \delta_{j}^{t}=\frac{\partial L}{\partial a_{j}^{t}}, \end{array}$$

(7) $$\begin{array}{c} \frac{\partial L}{\partial w_{ij}}=\overset{T}{\underset{t=1}{\sum }}\frac{\partial L}{\partial a_{j}^{t}}\frac{\partial a_{j}^{t}}{\partial w_{ij}}=\overset{T}{\underset{t=1}{\sum }}\delta_{j}^{t}b_{i}^{t}. \end{array}$$

The main formula given here is to calculate the cumulative residual of the hidden layer because the output layer is the same as the traditional BP neural network. There are two parts in formula (5): one receives the residual returned by the output layer at the current time shown in formula (6) and the other receives the residual returned by the hidden layer the next time shown in formula (7).

The article "Accounting Earnings and Economic Growth, Trends, and Challenges: A Bibliometric Approach" was published in 2022. Journal: Comput Intell Neurosci.

There is also a neural network model that has been mentioned by researchers in recent years, which is the extended short-term memory model (LSTM). The LSTM is derived from the recurrent neural network (RNN) model, first proposed by Hochreiter & Schmidhuber [15]. It has the characteristics of the RNN model and can use the memory unit to process data to enhance the learning ability of the model. In the LSTM model, the unit replaces the neuron in RNN, and its structure consists of three parts: input gate *i*_*t*_, output gate *o*_*t*_, and forget gate *f*_*t*_ as follows:

(8) $$\begin{array}{c} i_{t}=\sigma \left(w_{i}x_{t}+u_{i}h_{t-1}+b_{i}\right),\\ o_{t}=\sigma \left(w_{o}x_{t}+u_{o}h_{t-1}+b_{o}\right),\\ f_{t}=\sigma \left(w_{f}x_{t}+u_{f}h_{t-1}+b_{f}\right),\\ c_{t}=f_{t}*c_{t-1}+i_{t}*\;\tan\;h\left(w_{t}x_{t}+u_{t}h_{t-1}+b_{t}\right),\\ h_{t}=o_{t}*\;\tan\;h\left(c_{t}\right), \end{array}$$

where *x*_*t*_ is the input to the memory layer, *c*_*t*_ is the cell state, and *h*_*t*_ is the output of LSTM. The sigmoid function is used as the activation function in the network, *w* is the output gate weight, and *b* is the output gate bias vector.

Particle swarm optimization (PSO) was born to optimize complex numerical models. It is based on artificial life theory and evolutionary calculations. It has now been widely used in various fields. [16]. PSO has an inherent guidance method that allows it to obtain improved valuable data. It can help to minimize the key parameter, the weights of the network model, to improve the learning speed of the LSTM.

The article "Accounting Earnings and Economic Growth, Trends, and Challenges: A Bibliometric Approach" was published in 2022. Journal: Comput Intell Neurosci.

Based on the existing PSO-LSTM model, Liang et al. [17] proposed a prediction method for emerging research topics, predicting the future popularity score of research topics based on historical observations. Their model shows as follows:

(9) $$\begin{array}{c} {\text{AFD}}_{i}={\text{DF}}_{i}-\alpha *{\text{ADF}}_{i-1}, \end{array}$$

(10) $$\begin{array}{c} P_{i}=\text{In}\left({\text{AFD}}_{i}+\delta \right)*\frac{{\text{DF}}_{i}+\delta }{{\text{DF}}_{i-1}+\delta }. \end{array}$$

Use formula (9) to measure the annual frequency AFD_*i*_ of each term, based on the number of documents that contain specific terms, where DF_*i*_ represents the document frequency of a given term at time *i* and *α* is the attenuation factor range from 0 to 1. It set to 0.9, which is a moderate decay rate, halving the impact of the subject after 5 years. Then, calculate the annual growth rate of the subject through ((DF_*i*_+*δ*)/(DF_*i*−1_+*δ*)). Finally, the activity score *P*_*i*_ is calculated by combining the AFD_*i*_ as shown in formula (10). Research terms and their occur times are defined as a time series set, and the model is trained based on the historical series to make the model have predictive capabilities.

The present research will draw on the model of Liang et al. [17] to predict the future research direction of aggregate earnings.

## 3. Findings and Discussion in the Bibliometric Analysis

### 3.1. Usefulness of Earnings

#### 3.1.1. Yearly Publication and Citation Frequency

After manually excluding the completely unrelated fields, 251 publications were obtained on WoS and 282 on Scopus. We will first implement a bibliometric analysis of the earnings usefulness research. This step is to find the position of aggregate earning research in the current academic world and explore its macro development trend. We used the data we have collected to compare the annual publications (Figure 1).

Figure 1 shows that the earliest evidence found on WOS dates from 1968, and until 1990, the research intensity was very low. The number of papers started to increase in the late 1990s and is increasing. They have a solid upward trend, with almost identical results for both databases. We believe that the reason why the results of the two databases are basically the same is related to the economic crisis. Although we cannot quantify its impact, the economic environment is also one of the influencing factors. Simultaneously, although the two databases' results show large fluctuations during 2010–2019, both curves have an exponential upward trend. According to the trend, this research will arrive in the third stage in a few years, which is the consolidation of the body knowledge stage.

The article "Accounting Earnings and Economic Growth, Trends, and Challenges: A Bibliometric Approach" was published in 2022. Journal: Comput Intell Neurosci.

For the quartiles of these publications in both databases, we found that more nonimpact journal publications are included in WoS, 24% in WoS compared to only 4% in Scopus. Also, the proportion of Q1 journals in Scopus accounts for 52%, while in WoS, it is only 38%. Among the two databases, papers on this topic, published in high-impact Q1 and Q2 journals, account for the majority, 57% in WoS, and 81% in Scopus, proving the importance of this topic (see Table1).

Secondly, we analyze annual citations of the two databases. Because the documents included in the two databases are different, we can see in Figure 2 that the two databases have significant differences. In WoS, the number of citations shows a steady upward trend from beginning to end, while in Scopus,it was very active from 1995 to 2006, and then, it shows a steep decline. Moreover, the number of influential papers is less than that in WoS. Hence, Scopus influence in this field declined after 2006. We believe that Scopus research studies have more development potential, and the development of new research directions can provide more support for the field innovation and development.

#### 3.1.2. Term Co-occurrence Maps and Research Lines

This section will compare and analyze the term co-occurrence maps generated using the two databases, which can help us view the most commonly used terms in this field. We adjusted the co-occurrence threshold to 10 times and then in the 5,205 WoS terms got 107 meets. VOSviewer only keeps the top 60% terms by default, so we only get 64 terms to generate maps. For Scopus data, we used the same settings and in 5,518 terms got 123 meets. Finally, 74 generated terms are retained.

The term co-occurrence maps based on the WoS and Scopus results are shown in Figures 3 and 4 respectively. According to the threshold, these terms can only be displayed when they occur ten times or more. In other words, when scholars mention them often. The closer terms have a stronger connection, forming clusters. These clusters are the existing research lines in the research area. We set the map to density visualization to better observe the hotspots of terms and their clustering distribution. The results in both databases were determined by VOSviewer and resulted in three clusters.

By comparing the two databases' results, we can find that each cluster in the two databases in Figures 3 and 4 has its representative terms clustered in three main research lines identified in the usefulness earnings research.

However, if we specifically analyze each cluster co-occurrences terms in the map, we can also find that several hotspots are not the same. These different terms represent different research directions within the two databases. We found that the two research directions are simultaneous. However, there is no strong correlation between many terms in Scopus. The research on these topics is more independent and does not form a knowledge network, but it is more novel than WoS. Scopus research is in the early stage of scientific development, and basic theoretical research is currently occupying the mainstream; it can provide support for follow-up research, so Scopus has more significant development potential in this field.

The article "Accounting Earnings and Economic Growth, Trends, and Challenges: A Bibliometric Approach" was published in 2022. Journal: Comput Intell Neurosci.

This first cluster focuses on the capacity of the earnings to value the stock price. Cluster focus also includes forecasts of future earnings and stock movements, examining the ability of accounting earnings to predict the future. Research such as Dechow et al. [18] found that accounting earnings information can better predict future cash flows. Brown & Han [4] used a first-order autoregressive model to show a stable relationship between the earnings period and the quarterly report aggregate information to predict future earnings data.

Furthermore, Lev et al. [5] focused on accrued profits and examined the usefulness of accounting estimates of accrued profits in predicting future returns. They found that increased accrual accounting estimates harm future cash flow predictions. More recently, Nallareddy et al. [19] found that, in general, cash flow is more advantageous than earnings in predicting future cash flows. Some researchers have already developed research on future excess earnings. For example, He & Narayanamoorthy [7] found in their research that the quarter-over-quarter change in earnings growth has a solid ability to explain future excess returns.

The literature of cluster 2 focuses on the return performance. It also focuses on the usefulness of earnings in companies' contracts, including research on its performance. Researchers use earnings-based financial indicators to study firm performance and ultimately apply them to contracts, such as debt and salary contracts. Research studies such as Sloan [20] investigated the role of accounting earnings in executive compensation contracts. Beatty et al. [21] studied the conservative modifications associated with debt contracts, finding that companies with more conservative financial reports would be more likely to make conservative changes. Rhodes [6] studied the impact of implicit incentives provided by earnings-based debt contracts on CEO compensation contracts. Li [22] pointed out that those earnings-based contract indicators are closer to EBITDA-based performance indicators, while Dyreng et al. [23] affirmed that those performance indicators based on accounting earnings are not conservative when used in contracts. Also, Curtis et al. [8] studied the impact of using adjusted earnings for performance evaluation on compensation.

The article "Accounting Earnings and Economic Growth, Trends, and Challenges: A Bibliometric Approach" was published in 2022. Journal: Comput Intell Neurosci.

Cluster 3 literature prefers research on the company risk. Some researchers are analyzing financial risk indicators based on accounting earnings information. The accounting surplus is linked to lower financial risk and accounting deficit with greater financial risk. At the same time, others focus on their risk on earnings or earnings-based variables. DeYoung & Roland [24] found that earnings volatility contains information about the company risk. More recently, Shahchera & Noorbakhsh [25] believed that the research on risk and earnings should also consider the company size and type. They found that the bank size is negatively related to earnings volatility. Other researchers try to explain the company risks based on many financial indicators, usually based on Beaver et al. [26], which analyzed the capacity of financial indicators to explain the market beta to measure the market system risk. Following their idea, Agusman et al. [27] showed that the standard deviation of the return on assets and the loan loss reserve could be essential concerning the absolute risk. Khan [28] proved the correlation between risk indicators and accounting indicators.

However, according to the two databases' outputs, their hotspot co-occurrence terms are not the same, and there are some different terms in each research line. This phenomenon is that even if the research in the two databases is in the same field, the different topics that researchers are concerned with will lead to different co-occurring terms. Analyzing these different terms can help us find the different research directions of the two databases' documents.

On the one hand, with cluster 1, although both databases focus on the earnings predictions for the future, in WoS, the report and the correlation between them have received more attention, such as Brown & Han [4], while in Scopus, researchers like Lev et al. [5] are more interested in the earnings quality. On the other hand, in cluster 2, both databases show that this research line focuses on the earnings return. However, in WoS, the pricing, estimation, and contract have also received attention, such as Beatty et al. [21]. Some studies have also focused on the book value and corresponding value, like Sloan [20] in Scopus. Finally, in cluster 3, both databases show research about risk. However, in WoS, some research also discusses the influencing factors and implications, such as Khan [28], with other publications discussing this research line benefit and design methodology like Agusman et al. [27].

The article "Accounting Earnings and Economic Growth, Trends, and Challenges: A Bibliometric Approach" was published in 2022. Journal: Comput Intell Neurosci.

Besides, in Figures 3 and 4, we can see that the degree of correlation between many terms is not very high, which means that the research on these topics is more independent and has not formed a knowledge network. Also, Figure 4, cluster 1 and cluster 3 have a mixed part, which means that some Scopus publications discuss two research directions simultaneously, and the research has a higher degree of innovation. According to what we mentioned above, Scopus research is in the early scientific development stage in the research on the usefulness of earnings. Theoretical basic research is now dominant. These theoretical studies provide support for follow-up research, so Scopus has more development potential in this field.

### 3.2. Aggregate Earnings

The article hopes to find a place for “aggregate earnings” research. After searching the original literature, we found that these studies are usually included in the first cluster on future earnings predictions. Kothari et al. [29] discovered the heterogeneity of aggregate earnings and company-level accounting earnings, which caused a wave of research on aggregate-level accounting information. Aggregate earnings with macroinformation began to be discussed by researchers.

#### 3.2.1. Yearly Publication and Citation Frequency

This article already discovered that aggregate earnings research belongs to the first research line of earnings usefulness research (see section 3.1). After manually eliminating irrelevant fields, we obtained 74 publications on WoS and 94 publications on Scopus. This research will discuss its research status and future development trends in the two databases in this section. First, it compared the two databases' annual publications (Figure 5) and annual citations (Figure 6) on this topic. At the same time, the quartiles were also collected from two databases corresponding to these publications, as shown in Table 2.

It can be seen in Figure 5 that the earliest WoS research was published in 1987. Scopus results are slightly later than WoS. As the years pass, the numbers of publications in the two databases have remarkable similarities, as it happened with the research of earnings usefulness (see Figure 1).

Moreover, this lately developed topic has not been rapidly developed until recent years. According to Price's law [13], it has just entered the exponential growth stage from the precursor stage of scientific development, so we believe that this topic now has excellent development potential. Furthermore, its development curve becomes exponential, indicating that it will become a research hotspot in the following years.

The article "Accounting Earnings and Economic Growth, Trends, and Challenges: A Bibliometric Approach" was published in 2022. Journal: Comput Intell Neurosci.

According to Table 2, for the quartiles of these publications, we found that in the same situation as the research on earnings usefulness, WoS included 19% publications from nonimpact journals, which is more than Scopus 4% in the topic of aggregate earnings. In addition, in the collection of Scopus in recent years, the proportion of Q1 journals is more significant than that of WoS (54% vs 43%). Also, the high-impact Q1 and Q2 journals account for a large proportion of the two databases, which have 63% in WoS and 83% in Scopus.

In Figure 6, it can be seen that the behavior of the two databases is very different. In WoS, the number of citations shows a regular upward trend from the beginning, while in Scopus, this field was very active from 1997 to 2005, but the number of citations decreased steadily after 2005. The present research considers there might be two reasons for this phenomenon. From a macroperspective, as shown in Figure 2, after 2005, the number of citations of Scopus research in the usefulness of earnings field has generally shown a downward trend. The research on aggregate earnings is one of the research lines on the earnings usefulness, which leads to unified results. Secondly, according to the comparative analysis of the terms in Figure 4, Scopus research is more independent than WoS research. The development of new areas has not received attention yet, leading to a decline in citations.

#### 3.2.2. Term Co-occurrence Maps and Research Lines

As with the previous analysis on the usefulness of earnings, the present research will analyze the research lines on aggregate earnings through the two databases' term co-occurrence map. In this analysis, to better study the clustering of terms, it also uses binary counts to generate maps. For the term co-occurrence threshold, called critical value, which refers to the lowest or highest value that an effect can produce, because of the limitation of the number of terms, this research modifies it to 5. In the end, it got 53 meets in WoS 1525 terms. Similarly, VOSviewer, in order to ensure the results are meaningful, only keeps the most important top 60% of terms, so we only get 32 terms to generate maps. We use the same settings for Scopus data, and in 180 terms, we get 73 meets. Finally, 44 generated terms are retained.

Figure 7 shows the term co-occurrence map based on the WoS results, and Figure 8 shows the term co-occurrence map based on the Scopus results. We also use density visualization to see the clustering of terms. VOSvievier identified three clusters in the two databases' co-occurrence maps circled in the picture.

The clusters show the different research lines. We can find that the results of both databases show that there are three research lines. We compared the co-occurrence terms of these three clusters and found that they are very similar, showing that there are three main research lines for the research of aggregate earnings. However, the results are also not identical due to the different internal links between the two databases. According to the results in the two figures, smaller research directions are different. In cluster 1, “paper,” “value,” “sample,” and “role” are hot terms. The results of these two databases both show that this research line is related to value research and existing papers, such as Kothari et al. [29], Gkougkousi [30], and Berkman & Yang [31]. According to these same terms, most research tends to be theoretically exploratory. However, research in WoS also pays attention to traditional earnings management research within this research line, such as Patatoukas [32], while the Scopus results also focus on the composition and prediction of earnings, such as Berkman & Yang [31]. In particular, even though Patatoukas [32] is also in this topic of Scopus results, it is different from the indexed results of WoS value-related topics.

The article "Accounting Earnings and Economic Growth, Trends, and Challenges: A Bibliometric Approach" was published in 2022. Journal: Comput Intell Neurosci.

For cluster 2, hotspot terms are “component,” “time,” “stock return,” and “market.” Both databases show market and stock return research, such as Patatoukas [32] and Berkman & Yang [31]. Nevertheless, WoS also focuses on time and market, such as Kothari et al. [29] and Kang [33]; and Scopus focuses on effect and some financial indicators like Cready & Gurun [34] and Berkman & Yang [31].

Finally, for cluster 3, terms “aggregate,” “accounting,” “country,” and “conservatism” are of concern for researchers. Both database studies focus on the country, accounting, and conservatism. These terms show that this research line is about the relationship between the micro- and macrolevels, such as Shivakumar [35], Konchitchki & Patatoukas [9], and Sumiyana et al. [36]. However, there are no more small research branches in WoS, and Scopus also mentioned other research directions such as importance and aggregate earnings management such as Gallo et al. [37] and Ball et al. [10].

Since this topic is relatively new, neither database has much research, and most are duplicated. Based on the above results, some research involves multiple research lines simultaneously. That makes it impossible to analyze each research area as precisely as in section 3. Therefore, based on the two databases' results, we analyze and review those studies with high impact.

Corporate earnings information represents a company's earnings level, and the higher the earnings level, the higher the returns listed companies earnings can bring, which has been widely accepted by scholars. However, in some studies, researchers have discovered different phenomena. For example, in a study of the aggregate earnings of data from the US market, Kothari et al. [29] found that aggregate earnings are negatively correlated with stock market returns. They also pointed out that the negative correlation of the results is due to the discount rate. They believed that the increase in aggregate earnings could increase investors' expectations about interest rates. Gkougkousi [30] also reached a similar conclusion in his bond market-based research. That leads people to think that the aggregate-level of accounting information has unique information content, which has led to scholars' enthusiasm for the aggregate earnings.

The article "Accounting Earnings and Economic Growth, Trends, and Challenges: A Bibliometric Approach" was published in 2022. Journal: Comput Intell Neurosci.

Patatoukas [32] decomposed the stock market returns into expectations for future market interest rates, expectations for future cash flows, and market return expectations. He validated the view of Kothari et al. [29] that aggregate earnings are positively correlated with the expected interest rates and the expected future cash flows. Kang [33] studied the impact of aggregate earnings on oil prices. He found that aggregate earnings contained information about fluctuations in oil prices. The inherent policy uncertainty response has exacerbated the impact of oil shocks on earnings and returns.

Have some researchers focused on the relationship between the aggregate earnings and the macroeconomy to explain the relationship between the enterprise and the capital market. The study of Kothari et al. [29] shows that aggregate earnings are positively correlated with macroeconomic growth (industrial output, GDP, personal consumption) over the same period. Moreover, Shivakumar [35] studied the relationship between aggregate earnings changes and several future macroeconomic performances and found that aggregate earnings changes were positively correlated with inflation.

The study of Konchitchki & Patatoukas [9] shows that aggregate earnings growth is positively correlated with future nominal GDP growth rates, which can predict future economic growth, giving the aggregate earnings the ability to predict economic growth a given quarter. Moreover, Cready & Gurun [34] showed that the aggregate earnings changes reflect the future discount rate and inflation information. Patatoukas [32] also verified this fact with the GDP deflator representing inflation. Shivakumar & Urcan [38] focused on explaining the aggregate earnings forecasting ability, and they verified that the aggregate earnings have predictive power for inflation because it predicts investment demand. Aggregate earnings affect future inflation through investment. Gallo et al. [37] used monthly data and quarterly data to empirically study the correlation between aggregate earnings and economic policies from the micro- and macrolevels. They believe that monetary policy ensures inflation, employment, and output. The aggregate earnings are related to future monetary policy.

The article "Accounting Earnings and Economic Growth, Trends, and Challenges: A Bibliometric Approach" was published in 2022. Journal: Comput Intell Neurosci.

More recently, Ball et al. [10] focused on the smoothness of company-level earnings. They investigated whether the smoothness of earnings can increase companies' information contribution to the aggregate earnings in future GDP forecasting research. Furthermore, they found that aggregate earnings are more focused on companies with smoother earnings, making these companies' financial information more informative. Sumiyana et al. [36] tested the ability of aggregate earnings to predict GDP growth. They compared the results of multiple countries and found that aggregate earnings, operating income, operating cash flow, and accrued expenses can predict GDP growth in the following one and two years. The company earnings component is an excellent predictor of future GDP growth. Berkman & Yang [31] defined the aggregate analyst recommendation at a country level as the value-weighted average of the stocks of companies incorporated in that country. They found that this proposal also helps predict GDP and aggregate earnings changes.

The above literature shows that the aggregate earnings indicator is a comprehensive reflection of the company's horizontal earnings. The total income index reflects the profit information of the whole company and affects the stock market return and future macroeconomic activities. Nevertheless, in accounting, according to the data obtained in this research, the topic of aggregate earnings information has not received enough attention. Therefore, it is necessary to study aggregate earnings, as it has practical significance for predicting economic growth.

#### 3.2.3. Research Trends of the Aggregate Earnings Research

The development and future trends of the aggregate earnings research are compared below based on the terms of the two databases.

For WoS term development, most terms occurred in 2010–2015. Specifically, around 2005 or before, only “stock returns” and “information” had attracted the attention of researchers, such as Kothari et al. [29], while, from 2010 to 2015, most terms, such as “prices,” “information-content,” and “accruals,” have become the focus of attention of researchers, like Cready & Gurun [34].

From 2015 to 2020, that is, in recent years, the terms such as “affect market returns,” “guidance,” “investment,” and “announcement” first appeared in the research on aggregate earnings. Currently, researchers are paying more attention to research on aggregate earnings and investment. After that, keywords such as “quality,” “tax avoidance,” and “economic growth” became hotspots, which means that in recent years, researchers have paid greater attention to the relationship between aggregate earnings and macroeconomics, for example, Patatoukas [32], Gallo et al. [37], and Ball et al. [10].

The article "Accounting Earnings and Economic Growth, Trends, and Challenges: A Bibliometric Approach" was published in 2022. Journal: Comput Intell Neurosci.

For Scopus, the term development around 2005 or before, “employment,” “wage,” and “accrual” have attracted the attention of researchers. After 2005, research on the relationship between aggregate earnings and national economic growth began with “economic analysis” and “economic growth.” Moreover, till around 2020, “gross domestic product” has become the latest research hotspot [9,10].

Comparing the results in WoS and Scopus, the term “accrual” occurred in WoS around 2010, five years later than Scopus, showing that Scopus research has paid more attention to accrual accounting research earlier in this field. Furthermore, related research on “earnings management” occurred in WoS before 2015 and in Scopus not until 2015–2020. The study of earnings management belongs to the traditional study of earnings usefulness. Again, this is also why the “stock return” occurred in WoS earlier than 2005 and in Scopus not co-occurred until 2015–2020. However, the Scopus research on “economic growth” has occurred around 2015 and in WoS did not occur until recent years.

## 4. Findings and Discussion Applying the Network Model

To better investigate the RQ2 in this article, this article is based on the second part about the ARIMA forecasting model and neural network forecasting model theory to analyze the sample data of this research. The present research considers the ability of different prediction models to predict the terms activity score *P*_*i*_ in formula (10). Therefore, comparing the performance of the most common forecasting model ARIMA from financial modeling and the neural network model. This research splits the 1525 terms from WoS and 180 terms from Scopus into series with a fixed length of 5. The value of each series is the real value at the historical term occurrence time. First,the PSO-LSTM model of this study is trained using sample data and then compared the predictive capabilities of financial modeling and neural network models for terms. The results are shown in Table 3.

Through the longitudinal comparison of the ARIMA model and neural networks in the forecast, whether it is forecast, the MSE value, RMSE value, and MAE value of the ARIMA model are similar. Compared with the neural network model, it has different degrees of reduction most of the time. Among them, the indicators of the ARIMA model for the 5-year forecast part were reduced by 0.0504, -0.0031, and 0.0513. Indicators of the ARIMA model for the 10-year forecast part were reduced by 0.0612, -0.0336, and 0.0157. For the 20-year forecast part, the various indicators of the PSO-LSTM model of PSO were reduced by -0.0850, 0.0563, and 0.0556 in turn.

The article "Accounting Earnings and Economic Growth, Trends, and Challenges: A Bibliometric Approach" was published in 2022. Journal: Comput Intell Neurosci.

Then, according to the PSO algorithm, the present research selects mini-batches' learning size to 128, which can reduce the number of iterations and make the training of the model more efficient, and selects the epoch to 10, according to the total sample size, that is, 1705, so the iteration is 134. After completing the selection of the model parameters, the 1525 terms from WoS and 180 terms from the Scopus of training data are split into a fixed length of 5, and the data input dimension is 5. Then, the optimization algorithm model is constructed and trained. The results are shown in Table 4.

Through the longitudinal comparison of the ARIMA model and the optimized algorithm model in the forecast, whether it is forecast, the MSE value, RMSE value, and MAE value of the optimized algorithm model are almost all smaller than the ARIMA model. Among them, the indicators of the optimized algorithm model for the 5-year forecasting part decreased by 0.0134, 0.0650, and 0.0116. The indicators of the optimized algorithm model for the 10-year forecasting part decreased by 0.0594, 0.0325, and -0.0155. The indicators of the optimized algorithm model of the 20-year forecast part decreased by 0.0267, 0.0006, and 0.0242 in turn. It can be seen that the optimized algorithm model is indeed effective for the correction of the ARIMA model, and the hybrid model can achieve better prediction results.

Next, the present research imported the terms data of the two databases into the models (15) and (16), which the PSO-LSTM model of Liang et al. [17]. According to the prediction results of the model, the ranking of the influence of the two databases on the terms of this topic is shown in Table 5.

Hence, we find that traditional research on earnings will continue to receive attention, such as returns, stock market returns, and earnings quality. Some studies extend the usefulness of earnings research and have gathered attention from scholars. Although WoS has also begun to focus on economic development research in recent years, but economic growth period is very small and the loss of agglomeration, enterprises, funds, talents, technology, and other factors of production are absorbed by a larger center or economies, and there are not many related studies. Moreover, researchers will pay more attention to the research on tax avoidance. Also, more research will be combined with macroeconomic research in the near future of WoS research, whether direct research on macroeconomic indicators or macroeconomic forecasts.

The article "Accounting Earnings and Economic Growth, Trends, and Challenges: A Bibliometric Approach" was published in 2022. Journal: Comput Intell Neurosci.

By comparing the results, we are more concerned about economic development issues. We found that Scopus research will develop better than WoS research in terms of aggregate earnings in the future because macroeconomic terms are more active in Scopus. Hence, Scopus focus will no longer be too confined to the traditional earnings usefulness topics, allowing them to develop rapidly in new directions.

However, WoS research has slowly developed in the subject of macroeconomic development. And there is no vitality in future forecasts. Because most of it is limited to traditional research questions on aggregate earnings, most of its research ideas have been fully developed in WoS and are blocking the development of new topics.

## 5. Conclusions

Under the current complex and challenging economic background, accounting information has a greater impact on economic development.Most research on the usefulness of accounting information is directed at investors, creditors, and individuals from the current research status. At the same time, there is scarce research related to government and country macroeconomic policies. For the analysis and forecasting of GDP, there is a lack of research from an accounting perspective. Therefore, the present research contributes to narrowing this gap. The bibliometric analysis of the related research on aggregate earnings explores the relationship between the accounting income of microenterprises and the country macro-GDP.

For a better bibliometric analysis of aggregate earnings, we first analyzed the relevant research on the usefulness of earnings. In the comparative analysis of influence, the present research found that Scopus research has less impact than WoS. Moreover, comparing the term co-occurrence maps, we found that Scopus research topics are more independent, without forming a knowledge network, but more novel. Scopus development is still in the early stage of scientific development in this field and has more significant development potential. WoS research can clearly distinguish three different research lines, and there is no strong correlation between the three of them. At the same time, we believe that developing WoS research in this field will have significant resistance.

In the comparative analysis of the co-occurrence terms map, we found that there are not many publications in the two databases because the topic is relatively new. Moreover, some research involves multiple research directions. Due to a larger number of articles, WoS shows more terms. Nevertheless, in the development of new topics, Scopus performance is better than WoS, whose research in this field is still focused on the topic of traditional earnings usefulness research.

The article "Accounting Earnings and Economic Growth, Trends, and Challenges: A Bibliometric Approach" was published in 2022. Journal: Comput Intell Neurosci.

In the forecast of future research of aggregate earnings topic, we first compared the predictive capabilities of the traditional ARIMA model and neural network model and found that the optimization algorithm model performed best. We used it to predict the future active terms of the two databases. Overall, Scopus research developed better than WoS research in aggregate earnings research. Furthermore, in future development, it will have more potential, while WoS research in this field will gradually lose attention.

Although some researchers have obtained seemingly reliable results through theoretical and empirical research, these conclusions have many interfering factors, resulting in researchers' results not being unified. After determining the relationship between earnings and the country's economic growth, empirical research proves that using the methodology on aggregate earnings is correct and credible. Moreover, we have great expectations for exploring research on earnings data ability to predict future economic growth. In the future, empirical research using a more comprehensive range of samples will continue.

## Figures and Tables

**Figure 1:** The usefulness of earnings yearly number of publications in WoS and Scopus.

**Figure 2:** The usefulness of earnings yearly number of citations in WoS and Scopus.

**Figure 3:** WoS term co-occurrence map.

**Figure 4:** Scopus term co-occurrence map.

**Figure 5:** Aggregate earnings yearly number of publications in WoS and Scopus.

**Figure 6:** Aggregate earnings yearly number of citations in WoS and Scopus.

**Figure 7:** WoS term co-occurrence map.

**Figure 8:** Scopus term co-occurrence map.

**Table 1:** The usefulness of earnings publications' quartiles in WoS and Scopus.

	WoS						Scopus					
	Q1	Q2	Q3	Q4	Other	Total	Q1	Q2	Q3	Q4	Other	Total
1968	3					3						0
1976						0	1					1
1984						0	1					1
1985						0	1		1			2
1986						0	1					1
1987						0	2					2
1988			1			1		1	1			2
1989	2					2	1					1
1990						0		1				1
1992	3		1			4	1	2				3
1993	5	1				6	2	1				3
1994	1	2	1			4	2	2	2			6
1995	1					1	3	2				5
1996	2					2	4	1				5
1997		1				1	4	2				6
1998	1		1			2	5	2	1		1	9
1999				1		1	7	3	1			11
2000	2					2	2	2				4
2001	3	3				6	5	3		1	2	11
2002	6		1			7	4	4				8
2003	6					6	5	1			2	8
2004	4				3	7	4	2			1	7
2005	2					2	2	5				7
2006	3	1	1		2	7	8			2		10
2007	2	1	1		2	6	5	1	4	1	1	12
2008	2	1	1	1		5	5	4		1	1	11
2009	1	4	1		1	7	5	3	2			10
2010	6	1	4	1	1	13	8	4	1	1		14
2011	5	2	2	1	2	12	8	3	1			12
2012	5	3		1	3	12	7	9	2	1	2	21
2013	2	2	2	1	3	10	4	1	1			6
2014	4	5	1	2	1	13	6	2	1	2	1	12
2015	4	4	3		7	18	6	1	1	1		9
2016	6	6	4	1	8	25	11	6	1	4		22
2017	5	2	4	1	13	25	2	6	2	1		11
2018	4	3	1		6	14	8	4	3			15
2019	5	5	5	3	9	27	6	3	2	1		12
Percentage	0.38	0.19	0.14	0.05	0.24	251	0.52	0.29	0.10	0.06	0.04	282

The article "Accounting Earnings and Economic Growth, Trends, and Challenges: A Bibliometric Approach" was published in 2022. Journal: Comput Intell Neurosci.

**Table 2:** Aggregate earnings publications' quartiles in WoS and Scopus.

	WoS						Scopus					
	Q1	Q2	Q3	Q4	Other	Total	Q1	Q2	Q3	Q4	Other	Total
1987						0		2				2
1991						0		1				1
1992	1					1	1					1
1993						0	1					1
1995	1					1						0
1996	1					1	1					1
1997						0	1					1
1999		1				1	2	2				4
2001	1					1	1		1			2
2002	1					1	1	1				2
2003		1				1	1					1
2004	2					2	2		1			3
2005	2					2	2	2				4
2006	1	1				2	1	1				2
2007	2			1		3	3	2	1	1	1	8
2008	1	1	2	1	1	6	3	1	1		1	5
2009	2	1	1	1		5	4		1			5
2010	1	1				2	2	1				3
2011	1	2	1			4	4	1	1	1	1	8
2012		1				1	1					1
2013	1	1	1			3	2	1	1			4
2014	3	1				4	3	1	1		1	5
2015	2	2			3	7	2	2	1			5
2016	3	1	2		2	8	2	2				4
2017	2				1	3	2	1				3
2018		1	1		1	3	2	2	1			5
2019	4		2		6	12	6	4	2			12
Percentage	0.43	0.20	0.14	0.04	0.19	74	0.54	0.29	0.13	0.02	0.04	93

**Table 3:** Forecast effect comparison.

		Mean square error (MSE)	Root mean square error (RMSE)	Mean absolute deviation(MAE)
5-year forecast effect comparison	Neural networks	0.1787	0.4916	0.2853
	ARIMA model	0.2291	0.4885	0.3366

10-year forecast effect comparison	Neural networks	0.4790	0.7315	0.4739
	ARIMA model	0.5402	0.6979	0.4896

20-year forecast effect comparison	Neural networks	0.7440	0.7745	0.6899
	ARIMA model	0.6590	0.8308	0.7455

**Table 4:** Comparison of optimized forecasting effects.

		Mean square error (MSE)	Root mean square error (RMSE)	Mean absolute deviation (MAE)
5-year forecast effect comparison	Neural networks	0.2158	0.4574	0.3106
	ARIMA model	0.2227	0.5475	0.2739
	Optimization algorithm model	0.2093	0.4825	0.2623

10-year forecast effect comparison	Neural networks	0.4834	0.6987	0.5419
	ARIMA model	0.5422	0.7238	0.4509
	Optimization algorithm model	0.4828	0.6913	0.4664

20-year forecast effect comparison	Neural networks	0.6610	0.8358	0.6799
	ARIMA model	0.6744	0.7970	0.6684
	Optimization algorithm model	0.6477	0.7964	0.6442

**Table 5:** Forecast term ranking of two databases.

WoS ranking	Optimization algorithm model	Scopus ranking	Optimization algorithm model
1	Returns	1	Accruals
2	Accruals	2	Economic growth
3	Earnings quality	3	Economic analysis
4	Stock market returns	4	Returns
5	Economic growth	5	United State
6	Tax avoidance	6	Earnings management
7	Information content	7	GDP
8	Prices	8	Information
9	Earnings management	9	Wage
10	Announcement	10	Employment

The article "Accounting Earnings and Economic Growth, Trends, and Challenges: A Bibliometric Approach" was published in 2022. Journal: Comput Intell Neurosci.

## Data Availability

The data that support the findings of this study are available from the corresponding author upon reasonable request.
